# Design and Calibration of Torque Measurement System of Comprehensive Performance Test Instrument of Industrial Robot Reducer

**DOI:** 10.1155/2022/8155818

**Published:** 2022-02-01

**Authors:** Zhen Yu, Zurong Qiu, Hao Li, Jie Xue, Wenchuan Hu, Chenglin Wang

**Affiliations:** ^1^State Key Laboratory of Precision Measurement Technology and Instrument, Tianjin University, Tianjin 300072, China; ^2^Tianjin University of Technology and Education, Tianjin 300350, China; ^3^College of Mechanical Engineering, Tianjin University of Technology, Tianjin 300384, China

## Abstract

The measurement of input and output torque of a precision reducer, the core component of an industrial robot, plays a vital role in evaluating the robot's performance. The TMSIS and TMSOS of a vertical cylindrical high-precision reducer detector were designed and investigated in this study to realize the accurate measurement of input and output torque of the reducer. Because a transmission chain connects the torque transducer and the reducer, the characteristics of the inevitable additional torque are analyzed in detail. A torque calibration device is developed to realize the calibration of the torque measurement system. The readings of the torque calibration device are compared with the data of the instrument's torque measurement system to realize the instrument's torque calibration. The improved particle swarm optimization and Levenberg–Marquardt algorithm-based radial basis function neural network is used to compensate for the error of the torque measurement system. The parameters of the RBF neural network are settled according to the characteristics of the additional torque and the torque calibration results. The experimental results show that the torque measurement accuracy of the torque measurement system can reach 0.1% FS after torque calibration and error compensation.

## 1. Introduction

In recent years, as a transmission device, the reducer has had a wide range of applications in machinery and automation [1]. Particularly, as the critical component [2], the performance of a reducer directly affects the motion accuracy and efficiency of the entire robot transmission system [3]. Therefore, the performance detection of reducers considerably influences the development of robots and the entire manufacturing industry [4–6]. The performance parameters of the reducer generally include the no-load friction torque, torsional stiffness, and transmission efficiency [3, 7, 8]. Many scholars have extensively studied the optimization of the internal parts [9], overall structure [10], and dynamic performance of the reducer [11, 12]. However, these studies are limited by measurement means and equipment, which severely hinders the improvements to the reducer performance. Experts in related fields have studied the reducer testing equipment and made technological progress [13–15]. However, in terms of practical application, this equipment cannot meet the development need of robot precision reducers from practical application. The measuring equipment mainly needs to be improved [16, 17] in terms of instrument structure, torsional stiffness [18], error analysis, and precision traceability [19].

Figure 1 shows the structure of a commonly used reducer comprehensive performance tester. Because of the cantilever support structure and the guide rail, the torsional rigidity of the instrument is weak. The weak stiffness of the shaft causes torque fluctuation [20], adversely affecting the measurement accuracy of the instrument [21, 22]. Moreover, installing and disassembling the tested reducer takes more than an hour in practicality, severely complicating industrial applications [23].

The authors previously invented a vertical cylindrical worktable precision reducer comprehensive detector (Patent No.: 201910175593.8). Through the symmetry of the structure and the force closed design, the instrument effectively solved many problems, such as weak stiffness, complex deformation, and difficult precision traceability. However, the torque sensor on the test instrument and the reducer under test are installed in different locations, connected by a transmission chain between the two. The transmission chain will produce bending and torsion deformation in the measurement process, resulting in misalignment error. The misalignment error will lead to the bending moment [18], which consumes part of the torque transmitted by the shaft [24]. As a result, there is a deviation between the reducer's actual input and output torque and the instruments' torque sensor reading value [21,25]. We call this part of the torque deviation “additional torque.” Therefore, the measurement results of the torque sensor on the instrument cannot be used as the reducer's actual input and output torque [26–28].

The characteristics of the additional torque are analyzed in this paper. The applicable neural networks theory improvement has provided a good reference for solving this problem. Scholars have done much work on the optimization of the torque control system [29, 30] and optimal reparameterization in industrial cyber-physical systems (ICPSs) [31]. All the works above are well-established (fuzzy systems, MLP) and promising techniques that are good references for applying neural networks theory. Based on the features of the additional torque and the applicable neural networks theory, a new method of improving the torque measurement accuracy using the improved particle swarm optimization and Levenberg–Marquardt algorithm-based (IPSO-LM) radial basis function (RBF) neural network is presented to eliminate the influence of additional torque.

The contribution of this paper is the method of improving the torque measurement accuracy by the IPSO-LM-RBF neural network, which is not limited to the background of improving the torque measurement accuracy. A torque calibration device is developed to realize the calibration of the torque measurement system. The parameters of the IPSO-LM-RBF neural network are settled according to the characteristics of the additional torque and the torque calibration results. The proposed method focuses on improving our team's previously developed measurement device. It provides a reference for improving and applying the IPSO-LM-RBF neural network to the torque measurement area. Moreover, it also provides a reference for improving the measurement device developed previously.

## 2. Structure and Characteristics of Torque Measurement System

As shown in Figure 2, the instrument's structure is vertical, and its functional components are vertically connected in series. The device consists of five subsystems: the guide rail mechanism, torque measurement system on the input side (TMSIS), tested components (TC), torque measurement system on the output side (TMSOS), and workbench. The case body and the worktop compose the workbench, and the TMSOS fixed on the workbench extends from top to bottom. Driven by the guide rail mechanism, the TMSIS can move along the *Y* and *Z* directions, providing space for the reducer's installation and disassembly. Different types of tested reducers can be installed in the TC. The TC and the instrument are connected using standard positioning and mechanisms to form the TC.

As the core components of the instrument measurement system, the TMSIS and TMSOS are mainly composed of four parts: motor, torque transducer, test mode conversion components, and other connecting components. The TMSIS and TMSOS adopt a cylindrical structure, and the disc support ensures that the transmission shaft is located in the center of the cylinder. This design improves the instrument's stiffness, simplifies the device's deformation, and reduces the number of error sources. In addition, the test mode conversion structure is designed for the measurement shafting, which allows for the input or output shaft of the tested reducer to be in an unconstrained, driven, or locked state to meet the functional requirements of different dynamic and static performance tests. The structure of TMSIS and TMSOS is shown in Figures 3 and 4.

As described above, the cylindrical structure of the TMSIS and TMSOS improves the instrument's stiffness, simplifies the device's deformation, and reduces the number of error sources. Then, the characteristics of the TMSIS and TMSOS are described in detail as follows:

### 2.1. Minimum Deformation

Because of the force change, the TMSIS and TMSOS may have structural deformation or operation state change in the measurement process. These changes lead to torque fluctuation and affect the torque measurement accuracy. Therefore, the stiffness of the torque measurement system is improved to make its deformation as small as possible and thereby ensure high measurement accuracy. In most horizontal structures, discrete cantilever supports are placed on a horizontal platform to hold each series component.  Figure 5 shows the deformation of a cantilever bracket under torque. The coaxially between adjacent elements realized by the cantilever bracket is likely to be damaged under the deformation caused by measuring torque. The deformation of a horizontal test bench is shown in Figure 6. These deformations lead to torque fluctuation and reduction of the torque measurement accuracy. Even if the stiffener is added to the cantilever beam to improve the stiffness, it can only alleviate this shortcoming to a certain extent. It cannot change the low stiffness of the instrument in essence.

The torque measurement system described in this study adopts a vertical cylindrical structure with disk support inside. Each part of the shafting is supported by a disc fixed in a vertical hollow cylinder. Therefore, the gravity of the drive shaft does not affect the alignment of the shafting. The transmission shaft transmits torque to the hollow cylinder through the disc plate in the measurement. The torque is transmitted to the hollow cylinder along the circumferential direction, and the uniform force characteristics improve the stiffness of the torque measurement system. At the same time, the cylinder and the tested reducer are used to form an axisymmetric spatial torque closed structure, thereby making the measured torque an “internal force.” The guide rail structure is separated from the measured torque ring to improve the system's stiffness. The deformation of the torque measurement system shell under torque is shown in Figure 7. The comparison of Figures 6 and 7 shows that when bearing the same torque and the overall dimensions are the same, the shell deformation of the torque measurement system is less than that of the horizontal structure. The instrument used in this study significantly improves the overall stiffness of the mechanism. At the same time, the cylindrical worktable makes the materials distributed in a ring, and the structure maximizes the torsional stiffness obtained by the same volume of materials.

### 2.2. Minimum Misalignment Error Based on Common reference Axis

Misalignment error refers to the relative position error between two parts of the connecting elements, i.e., the installation position error between two separate parts. The misalignment error of series components leads to the bending and torsional deformation of the shaft. As the deformation changes the stress state of the bearing part, the additional torque is included in the measurement results. In the traditional horizontal structure, the complex structure and easy deformation of the cantilever support complicate the quick alignment of various parts of the shaft system and the alignment of the tested reducer and the shaft system. As each component is an elastomer in dynamic measurement, the complex deformation causes complex additional torque, unfavorable for torque measurement.

Therefore, the torque measurement system of the vertical cylindrical detector adopts the installation reference axis of the tested reducer as the measurement reference axis of the instrument. Moreover, the gravity direction of each component is along the axis direction to reduce the influence of gravity. Another essential feature of the cylindrical worktable is that the deformation shape is simple. The disc support's radial symmetry is conducive to ensuring the accurate alignment of each axis on the measuring shafting. The additional torque caused by the deformation is easy to compensate accurately.

### 2.3. Synchronous Acquisition

In the performance index of the reducer, torque is the critical factor. Torque fluctuation affects the measurement accuracy to a certain extent. The fluctuation torque often presents a nonlinear relationship between the input and output torque of the tested reducer. Therefore, the synchronous acquisition of the TMSIS and TMSOS torque signals must be emphasized. Otherwise, the data at different times are not comparable and cannot effectively reflect the actual state of the transmission characteristics of the tested reducer. Hence, the torque signals of the TMSIS and TMSOS are input from the same interface of the acquisition system, collected under the same clock, aligned one by one according to the time mark, and stored in the same file.

The torque measurement system designed in this study adopts a strain torque transducer, and the output signal is a frequency signal based on the 422 communication protocol. Through the FPGA programmable module of the data acquisition system, the frequency signals of the TMSIS and TMSOS are collected synchronously. Then, the frequency signals are transmitted to the computer. The computer converts the torque signal according to the corresponding relationship between frequency and torque. Through this method, the data of multiple torque transducers can be collected synchronously. The corresponding relationship between frequency and torque is as follows:

(1) $$\begin{array}{c} T=\frac{f-f_{e}}{f_{p}-f_{e}}\times N\left(\text{when }f>f_{e}\right),\\ T=\frac{f_{e}-f}{f_{e}-f_{r}}\times N\left(\text{when }f>f_{e}\right). \end{array}$$

In the equations above, *f* is the frequency, *T* is the torque, *f*_*e*_ is the zero point of the frequency, *f*_*p*_ is the maximum value of the frequency, and *f*_*r*_ is the minimum value of the frequency.

## 3. The Analysis of the Additional Torque

Although the designed vertical cylindrical precision reducer detector has many advantages, the torque transducer in the instrument and the reducer under test are connected by a transmission chain between the two. Thus, because of the influence of the inevitable additional torque, the measurement results of the torque transducers also cannot be considered to be the actual input and output torque of the reducer. The additional torque at this apparatus can also be included in the measurement results of other test systems using the same transmission chain between the torque sensor and the reducer. The causing of the additional torque is analyzed in detail in the following sections using TMSIS as an example.

Many factors result in uneven frictional forces around them [14, 24, 25]. The uneven frictional forces can lead to the consumption of the torque of the transmission system, which is the additional torque.  Figure 8 shows a bearing, spline sleeve, and spline shaft (in blue) between the torque transducer and the tested reducer when the TC is placed at the test location. The following section analyzes the three main parts of the additional torques.

### 3.1. Additional Torque due to Friction at Bearings

Irrespective of the type of bearing, friction torque is mainly composed of two kinds of torque [32]. The first one is the torque related to the structures of bearings and the property of lubricating oil. The second one is the torque related to the material of the bearings and the torque transmitted by the shaft. The expression of the components of friction torque Δ*T*_1_ is shown in the following equation.

(2) $$\begin{array}{c} {\mathrm{\Delta T}}_{1}{=\text{M}}_{0}{+\text{M}}_{1}. \end{array}$$

In the function, *M*_0_ is the torque related to bearings' structures and the property of lubricating oil in N·mm. *M*_1_ is the torque related to the material of the bearings and the torque transmitted by the shaft in N·mm.

The torque related to the structures of bearings and the property of lubricating oil can be expressed as follows [32]:

(3) $$\begin{array}{c} {\text{M}}_{\text{0}}{=160\times 10}^{-7}{\text{f}}_{\text{0}}D_{m}^{3}. \end{array}$$

where *D*_*m*_ is the average diameter of the bearing in mm, *f*_0_ is the parameter related to the structures of bearings, and the lubrication conditions in N/mm^2^.

The torque related to bearings' material and the torque transmitted by the shaft can be expressed as follows [32]:

(4) $$\begin{array}{c} M_{1}=f_{1}P_{1}D_{m}=\frac{f_{1}TD_{m}}{r}, \end{array}$$

where *f*_1_ is the friction parameter related to the material of the bearings and the torque transmitted by the shaft, *P*_1_ is the bearing load in N, *T* is the torque transmitted by the shaft in N·mm, and *r* is the shaft radius in mm.

### 3.2. Additional Torque Caused by Bending Related to Misalignment Errors

The spline sleeve and spline shaft play a significant role in TMSIS. Under ideal working conditions, the central axis of the torque transducer and the tested robot reducers should be oriented along the same central line. However, in actual production, this ideal situation does not exist. Manufacturing errors in the components and assembling errors often lead to deviations of the axle center-line. The status of the radial misalignment that exists between the torque transducer shaft and the tested robot reducer is shown in Figure 9.

In Figure 9, O1Z1 represents the axis of the torque transducer in TMSIS and O2Z2 represents the axis of the input shaft of the tested robot reducer. ∆*X* represents the offset between O2Z2 and O1Z1 axes in the radial direction. When a radial error ∆*X* exists, the torque measured by the torque transducer, which is also the torque transmitted by the shaft, corresponds to the combination of bending moment and torque. The torque transferred to the tested robot reducer is lower than that measured by the torque transducer. The additional torque caused by bending related to the radial error is given by [33],

(5) $$\begin{array}{c} \mathrm{\Delta T}2=\text{ KL}\left(\mathrm{\Delta X}+\frac{\text{T}}{\mathrm{r\varepsilon}}\right), \end{array}$$

where *K* is the coupling elastic coefficient, ∆*X* is the radial error of the shaft, *r* is the shaft radius, *L* is the distance between the torque transducer and the tested robot reducer, ε is the strain coefficient, and *T* denotes the torque transmitted by the shaft.

The misalignment error consists of radial and angular displacements. The status of the angular misalignment between the torque transducer in TMSIS and the tested robot reducer is shown in Figure 10.

In Figure 10, O1Z1 represents the axis of the torque transducer in TMSIS and O2Z2 represents the axis of the input shaft of the tested robot reducer. ∆θ represents the angular misalignment error between the axes.

When an angular misalignment error exists, the torque measured by the transducer, which is also the torque transmitted by the shaft, represents the bending moment and torque combination. Therefore, the torque transferred to the tested robot reducer is smaller than that measured by the torque transducer. The additional torque because of bending related to the angular misalignment error is given by [33],

(6) $$\begin{array}{c} \Delta \frac{1}{2}\text{T}3=\text{T}\left(\text{cos}\Delta \theta -1\right)+\frac{\mathrm{Tcos\Delta \theta L}}{\text{r}}\text{.} \end{array}$$

where ∆θ is the angular misalignment error.

### 3.3. Additional Torque Caused by Compression of the Spline Coupling

An involute spline coupling is used in TMSIS to transmit the torque. The spline coupling engagement consumes part of the transmitted torque because of many factors, such as bending and compression [34]. The additional torque caused by bending is analyzed in the previous section. The additional torque caused by the compression of the spline coupling is analyzed in the subsequent sections.

Under Hertz contact condition [35], the relationship between contact pressure and indentation depth is as follows:

(7) $$\begin{array}{c} \alpha =\sqrt[{3}]{\frac{9\pi^{2}}{16}}\frac{P^{2}{\left(k_{1}+k_{2}\right)}^{2}\left(R_{1}+R_{2}\right)}{R_{1}R_{2}}. \end{array}$$

In the equation above, *α* is the indentation depth, *P* is the contact pressure, *R*_1_ is the radius of the spline sleeve, *R*_2_ is the radius of the spline shaft, *k*_1_ is the elastic coefficient of the spline sleeve, and *k*_2_ is the elastic coefficient of the spline shaft.

(8) $$\begin{array}{c} {\text{c}}_{\phi }=\frac{\text{P}}{\alpha }\text{,}\\ \text{P}=\frac{\text{T}}{{\text{R}}_{1}}\text{.} \end{array}$$

In the equation above, *c*_*ϕ*_ is the meshing stiffness of the spline coupling considered to be a constant.

Hence, the additional torque can be expressed as follows [34]:

(9) $$\begin{array}{c} {\mathrm{\Delta T}}_{4}={\text{T}-\text{T}}_{\text{i}}\\ {=\text{C}}_{\text{f}}\left(\phi_{\text{e}}{-\phi }_{\text{i}}\right)\\ =\frac{\text{T}\left(\phi_{\text{e}}{-\phi }_{\text{i}}\right)}{{\text{R}}_{1}\alpha }\\ =\frac{\text{T}\left(\phi_{\text{e}}{-\phi }_{\text{i}}\right)}{{\text{R}}_{1}}\sqrt{\frac{{\text{T}}^{2}{\left({\text{k}}_{1}{+\text{k}}_{2}\right)}^{2}\left({\text{R}}_{1}{+\text{R}}_{2}\right)}{{\text{R}}_{1}^{3}{\text{R}}_{2}}}\\ =\left(\phi_{\text{e}}{-\phi }_{\text{i}}\right)\sqrt{\frac{16}{{9\pi }^{2}}\frac{{\text{TR}}_{2}}{{\left({\text{k}}_{1}{+\text{k}}_{2}\right)}^{2}\left({\text{R}}_{1}{+\text{R}}_{2}\right)}}\text{.} \end{array}$$

*T*_*i*_ is the shaft torque, and *ϕ*_*i*_ and *ϕ*_*e*_ are the twisting angles for the spline shaft and spline sleeve.

By combining formulae (3)–(11), the additional torque *T*′ caused by the combined influence of the factors above can be obtained as follows:

(10) $$\begin{array}{c} {\text{T}}^{\prime }={\mathrm{\Delta T}}_{1}{+\mathrm{\Delta T}}_{2}{+\mathrm{\Delta T}}_{3}{+\mathrm{\Delta T}}_{4}\\ {=160\times 10}^{-7}{\text{f}}_{\text{0}}D_{m}^{3}+\frac{{\text{f}}_{1}{\text{TD}}_{\text{m}}}{\text{r}}+\text{KL}\left(\mathrm{\Delta X}+\frac{\text{T}}{\mathrm{r\varepsilon}}\right)+\text{T}\left(\text{cos}\Delta \theta -1\right)+\frac{\mathrm{Tcos}\mathrm{\Delta \theta L}}{\text{r}+\left(\phi_{\text{e}}{-\phi }_{\text{i}}\right)}\sqrt[{3}]{\frac{16}{{9\pi }^{2}}\frac{{\text{TR}}_{2}}{{\left({\text{k}}_{1}{+\text{k}}_{2}\right)}^{2}\left({\text{R}}_{1}{+\text{R}}_{2}\right)}}. \end{array}$$

Since the torque measured by the torque transducer is equal to the torque transmitted by the torque transducer shaft, we can conclude that the additional torque is no-linear dependent on the torque transmitted by the shaft.

## 4. Torque Calibration and Error Compensation

TMSIS and TMSOS adopt the serial and vertical arrangement of the multilevel parts. As one of the series links, the torque sensor is the core component of the instrument, and the measured torque value is a significant physical quantity representing the performance of the reducer. Therefore, the calibration of the torque sensor is essential. The existing calibration methods directly measure the output end of the torque sensor [36]. However, as is analyzed above, the friction at bearings, bending related to misalignment errors, and compression of the spline coupling produce additional torque. Therefore, there is a deviation between the reducer's actual input and output torque and the torque sensor's reading value. Therefore, it is necessary to calibrate the measurement results of TMSIS and TMSOS.

### 4.1. Torque Calibration Method

Comparing the known high-precision standard torque with the measurement result of the torque measurement system is a common calibration concept. Considering that the main torque measurement error originates from the additional torque, the calibration goal is to eliminate the influence of the additional torque on the measurement results. Therefore, a high-precision torque calibrator is proposed in this study, as shown in Figure 11. The calibrator comprises two high-precision torque transducers to calibrate the TMSIS and TMSOS. The external interface of the torque calibrator is the same as TC and can be connected with the instrument according to the standard interface. The torque calibrator is placed on the test station instead of TC during calibration. The upper and lower flanges of the torque calibrator are connected with the TMSIS and TMSOS, respectively, and pressed by a hydraulic mechanism. Then, the two torque measurement systems are calibrated, respectively. Because of the instrument's accuracy and stability of motor loading, when the torque calibrator is used to calibrate the torque measurement system in the device, 50 torque points evenly distributed in the whole range are selected for calibration, and the load torque needs to be filtered.

When the motor loads the torque, the readings of the torque measurement system and the torque calibrator are recorded simultaneously. By comparing the readings of the torque transducer in the calibrator, which are regarded as the standard torque, with the readings of the corresponding torque transducer in TMSIS and TMSOS, the real-time calibration data of the torque measurement system can be obtained. The specific process of torque calibration is shown in Figure 12.

### 4.2. Error Compensation Method

The causes of the additional torque are complex, and the number of points that can be calibrated is limited. Suppose the error compensation model of the torque measurement system can be constructed according to the 50 groups of scattered points calibrated by the torque calibrator and the error of the torque measurement system can be continuously compensated within the measurement range. Such a case would strengthen the guarantee of the instrument. Therefore, the radial basis function (RBF) neural network is used to approach any function with arbitrary accuracy, make full use of discrete calibration points, and realize continuous difference compensation in the measurement range.

As shown in Figure 13, the RBF neural network for torque measurement error compensation is a three-layer unidirectional propagation network. The RBF neural network comprises the input, output, and hidden layers. The three-layer RBF neural network can accurately realize any relationship between the input and output. This method can effectively simulate the relationship between the measurement results of the torque measurement system and standard torque tested by the torque calibrator. The parameters of the RBF neural network are settled according to the characteristics of the additional torque, the measurement results of the torque measurement system, and standard torque tested by the torque calibrator. There is one node in the network's input layer, which uses the measurement results of the torque transducer in the torque measurement system, represented by *T*_*i*_. There is one node in the output layer, expressed as *T*'*i*. The standard torque value is used as the output layer node. The 50 groups of scattered points, within the measurement range, calibrated by the torque calibrator are used to train the RBF neural network. The number of nodes in the hidden layer is automatically calculated and set by the Newrbe function. Repeated debugging shows that the RBF neural network converges the fastest with 50 nodes in the hidden layer, and the fitting effect is optimal. Therefore, it is determined that there are 50 nodes in the hidden layer, represented by *R*_*i*_. The weight from *T*_*i*_ to *R*_*i*_ is uik, using the relationship between the additional torque and the torque transmitted by the shaft shown in equation (10). The input signal is transformed by the function shown in equation (10) and sent to the hidden layer. The hidden layer unit is transformed by the radial basis function and sent to the output layer. The radial basis function is the Gaussian basis function. The weight from *R*_*i*_ to *T*'*i* is *W*_*ik*_, using a linear function as a function of the output layer. In the RBF function, the spread value of the expansion coefficient is the most critical parameter that size significantly impacts the RBF radial neural network [37]. In this study, the spread value is determined as 17 by the trial and error method.

The measurement results of the torque transducers in the torque measurement systems and the corresponding standard torque values are used as the learning samples for training. The output of the hidden layer is expressed as follows:

(11) $$\begin{array}{c} R_{i}=e^{-\frac{\left\|u_{ik}T_{i}-c_{i}\right\|}{2\sigma_{i}^{2}}}=e^{-\frac{\left\|\left(T_{i}-160\times 10^{-7}f_{0}D_{m}^{3}-f_{i}T_{i}D_{m}/r-KL\left(\Delta X+T_{i}/r\varepsilon \right)-T_{i}\left(COS\Delta \theta -1\right)/r-\left(\phi_{e}-\phi_{i}\right)\sqrt[{3}]{16/9\pi^{2}T_{i}R_{2}/{\left(k_{1}+k_{2}\right)}^{2}\left(R_{1}+R_{2}\right)}\right)-C_{i}\right\|}{2\sigma_{i}^{2}}}. \end{array}$$

In the equations above, *c*_*i*_ is the center of the i^th^ hidden layer node, σ_*i*_ is the width of radial basis function, and ‖·‖ is the Euclid Norm. The values of the center ci and width σ_*i*_ are calculated in the training of the hidden layer. The model of the output layer node is expressed as follows:

(12) $$\begin{array}{c} {{\text{T}}^{\prime }}_{\text{i}}=\sum_{\text{k}=1}^{50}{\text{W}}_{\text{ik}}{\text{R}}_{\text{i}}\text{.} \end{array}$$

In the equations above, *w*_*ik*_ denotes the output weights from *R*_*i*_ to *T*'*i*. The weights are calculated in the training of the last layer. The total error calculation function is expressed as follows:

(13) $$\begin{array}{c} \text{e}=\sum_{\text{i}=\text{k}}^{\text{n}}\sum_{\text{k}=1}^{50}{\left({{\text{T}}^{\prime }}_{\text{ik}}{-\text{t}}_{\text{ik}}\right)}^{2}, \end{array}$$

Here, *t*_*ik*_ denotes the calculation result of the output layer node. The structure and parameters of the RBF neural network can be acquired by adjusting the weights and thresholds. The trained RBF neural network can compensate for the errors of the torque transducer with more optimized fitting effects.

### 4.3. Calculation of Optimal Solution Based on IPSO-LM Algorithm

Among the RBF neural network parameters, *c*_*i*_, σ_*i*_, and *w*_*ik*_ must be determined by learning and training. The IPSO-LM algorithm is used to optimize the network parameters of the RBF neural network used in this study. The IPSO-LM algorithm combines the improved particle swarm optimization (IPSO) and Levenberg–Marquardt (LM) algorithms. Using the IPSO algorithm and LM algorithm to optimize the parameters of the RBF neural network can not only improve the prediction accuracy and make the prediction value more accurate but also reduce the running time of the algorithm.

In the IPSO algorithm, each particle represents a solution. The best solution among all solutions is the position of food. Each particle will look for the position of food in this region, and each particle will get its own position closest to the food in the process of looking for food. This position is called extreme individual value. The best position that all particles will get in the search process is the global extremum. Through these two positions, these particles will constantly adjust their speed and direction to approach the position of the food. The particle updates the speed and position of each particle through these two extreme positions. The update formula of particle velocity and position is as follows:

(14) $$\begin{array}{c} {\text{v}}_{\text{ij}}^{\text{m}+1}{=\text{WV}}_{\text{ij}}^{\text{m}}{+\text{C}}_{1}{\text{r}}_{1}\left({\text{P}}_{\text{ij}}^{\text{m}}{-\text{X}}_{\text{ij}}^{\text{m}}\right){+\text{C}}_{2}{\text{r}}_{2}\left(g_{j}^{\text{m}}{-\text{X}}_{\text{ij}}^{\text{m}}\right), \end{array}$$

(15) $$\begin{array}{c} {\text{X}}_{\text{ij}}^{\text{m}+1}{=\text{X}}_{\text{ij}}^{\text{m}}{+\text{lvX}}_{\text{ij}}^{\text{m}+1}, \end{array}$$

In the equations above, *i* = 1, 2,…, *n*, *j* = 1, 2,…, *J*, *m* = 1, 2,…, *M*, *m* is the iteration number. X_*ij*_^m^ is the position of particle *i* in space. *V*_*ij*_^*m*^ is the velocity of particle *i* in space. *c*_1_ and *c*_2_ are acceleration factors, usually *c*_1_ = *c*_2_. *r*_1_ and *r*_2_ are random numbers in the interval [O, 1], and *w* is the weight.

(16) $$\begin{array}{c} \text{w}=w\text{ max}-\left(w\text{ max}-w\text{ min}\right)\times \frac{\text{m}}{\text{m max}}. \end{array}$$

In the equations above, *m*_max_ is the maximum number of iteration, and *w*_max_ and *w*_min_ represent the maximum and minimum weights.

LM algorithm is a combination of gradient descent method and Gauss–Newton method. LM algorithm uses approximate second derivative information, requires less iteration time, converges very quickly, has good stability, and avoids falling into a local minimum. The iterative formula is as follows:

(17) $$\begin{array}{c} {\text{q}}_{m+1}{=\text{q}}_{m}-{\left(A_{M}^{T}{\text{A}}_{m}+\mathrm{\mu I}\right)}^{-1}A_{m}^{T}{\text{e}}_{m}\text{.} \end{array}$$

In the equations above, q_*m*_ is the control input sequence at the *m*^th^ iteration, q_*m*+1_ is the control input sequence at the next iteration, *μ* is the scale factor, *e*_*m*_ is the error between the predicted value of the network and the actual value, which can be obtained through (13), and A_*m*_ is the Jacobian matrix.

(18) $$\begin{array}{c} A_{m}=\left[\begin{array}{ccc} \frac{\partial e_{1}\left(q_{m}\right)}{\partial q_{1}} & \cdots & \frac{\partial e_{1}\left(q_{m}\right)}{\partial q_{n}}\\ \vdots & \ddots & \vdots \\ \frac{\partial e_{m}\left(q_{m}\right)}{\partial q_{1}} & \cdots & \frac{\partial e_{m}\left(q_{m}\right)}{\partial q_{1}} \end{array}\right]. \end{array}$$

The IPSO algorithm solves the objective performance function to obtain the optimal population solution's optimal control quantity result. The IPSO-LM algorithm takes advantage of the fast convergence speed and high search accuracy of the LM algorithm when it is close to the local minimum and the global fast convergence ability of the IPSO algorithm. It overcomes the disadvantage that the LM algorithm is too dependent on the initial value, and the IPSO algorithm is easy to fall into the local extremum. Taking the result of the IPSO algorithm as the initial value of the LM algorithm, the suitable optimal solution, i.e., the optimal control quantity, is obtained repeatedly. The algorithm steps are as follows:

1. Initialize the particle swarm optimization parameters and set the control quantity q_*m*_ as the initial particle. Set the current optimal position of each particle p_i_ and the current optimal position of all particles g, i.e., g  =  p_i_min__.
2. Update the speed and position of particles according to equations (14) and (15), calculate the fitness value of each particle, and record the extreme individual value p_i_ and the group extreme value g.
3. Compare the current position of each particle with p_i_. If it is better than p_i_, then update p_i_, otherwise let p_i_ be the same.
4. Compare the current p_i_ of each particle with g. If it is better than p_i_, then update p_i_. Otherwise, p_i_ remains unchanged.
5. If the termination condition is satisfied and the maximum number of iterations is reached, the iteration is terminated. Moreover, g is the optimal group solution, i.e., the current optimal control quantity. Otherwise, return to step 2.
6. Given the allowable training error values *e*, adjustment coefficient *β*, and the scale factor *μ*. Let *m* = 0, *μ* = 10^−4^, *β* = 10, and *e* = 10^−8^. The group optimal solution *g* obtained by the IPSO algorithm is taken as the initial value of the LM algorithm.
7. Calculate the control input sequence at the (*m* + 1)^th^ iteration *q*_*m*+1_ by equation (17).
8. Calculate the Jacobian matrix A_m_ by equation (18), and calculate the error e_m_ between the predicted value of the network and the actual value by equations (12) and (13).
9. If e_m_ < *e*, q_m_ is the optimal control quantity, go to step 11. Otherwise, take *q*_*m*+1_ as the new initial value to calculate the error-index function e_m+1_=q_m+1_e_m_.
10. If e_m+1_ < e_m_, let *k* = *k* + 1, *μ* = *μ*/*β*, return to step 7. Otherwise, the control quantity will not be updated, and hence, let q_m+1_  =  q_m_, *μ* = *μβ*.
11. Stop.

## 5. Experiment and Result

The torque calibration system was built according to the characteristics of the additional torque and the torque calibration and error compensation method described in the third and fourth sections.  Figure 14 shows the torque calibration experiment of the instrument. The torque calibration experiments were conducted to improve torque measurement accuracy. The torque calibrator was installed on the instrument for the calibration experiment. In the calibration experiment, the outputs of the torque transducers in the torque measurement systems, when there was no load, were adjusted to 0 Nm. The motor synchronously loaded the torque to the torque calibrator and the torque measurement system.

### 5.1. Torque Calibration and Error Curve Fitting

In calibration, the torque calibrator's standard torque and the torque transducers' readings in the torque measurement systems were recorded simultaneously. The full-torque error curve was obtained by training the RBF neural network according to the standard torque and the readings of the torque transducers in the torque measurement systems. The IPSO-LM algorithm was used to optimize the network parameters of the constructed RBF neural network. The population size of the IPSO algorithm was set to 50, the acceleration factors *c*_1_ = *c*_2_ = 2, *w* was dynamically updated by equation (18), *r*_1_ = 0.5, and *r*_2_ = 0.6. Since the selection of iteration times affected the training time, the maximum iteration time was preset to 1000. It was found in the training that the fitness curve of the IPSO algorithm had been stable when it was iterated 300 times. Hence, the maximum number of iterations was set to 300 times. The allowable error value of the LM algorithm was set to 10^−8^. The scale factor *μ* was 10^−4^. The adjustment coefficient *β* was 10. A total of 60 groups of data were obtained in the torque calibration experiment. In the experiment, the first 50 groups of data were selected for training the IPSO-LM-RBF neural network, and the remaining ten groups of data were used for testing. The appropriate error curves of TMSIS and TMSOS using the IPSO-LM-RBF neural network are shown in Figure 15 and 16. From these curves, the error compensation values of TMSIS and TMSOS at any torque are obtained.

### 5.2. Verification of the Torque Calibration and Error Compensation Method

The compensation effect of additional torque in the instrument using the proposed IPSO-LM-RBF neural network was verified using the remaining ten groups of data, and the torque measurement accuracy of TMSIS and TMSOS was determined. The torque measurement range of TMSIS was ±50 N·m, and the torque measurement range of TMSOS was ±2000 N·m. Positive and negative indicate loading in the clockwise or counterclockwise direction. We selected 50 sampling points in the full range for comparative analysis. The torque measurement errors of TMSIS and TMSOS before and after error compensation are shown in Figures 17 and 18, respectively. The results show that the maximum error of TMSIS is 0.045 N·m (0.9‰FS), and the maximum error of the TMSOS is 1.9 N·m (0.95‰FS). The repeatability of the torque measurement results after error compensation was obtained using the remaining ten groups of data. Three groups of experimental data at TMSIS and TMSOS are shown in Tables 1 and 2, respectively. By error compensation, the torque measurement accuracy of TMSIS and TMSOS can reach 1‰FS. For comparison, polynomial fitting and BP neural network were used to compensate for the error of the torque measurement system, respectively. The torque measurement error of TMSOS after compensation is shown in Figure 19.

### 5.3. Comprehensive Uncertainty

As the comparison method is used in the calibration of TMSIS and TMSOS in the instrument, the sources of uncertainty mainly include the measurement error of TMSIS and TMSOS, the possible data drift of the torque transducers, the random error caused by fluctuation of load, and measurement error of the torque calibrator.

The first component of uncertainty, *U*_1_, is caused by the measurement error of the torque transducer in the torque measurement system. According to the test report provided by the German metrology institute, when the torque transducer leaves the factory, the uncertainty of this part is *U*_1_ = ±0.05% FS.

The second component of uncertainty, *U*_2_, is caused by the possible data drift of the torque transducer from the last calibration owing to temperature changes. According to the instructions of the torque transducer, the uncertainty of this part is: *U*_2_ = ±0.02% FS.

The third component of uncertainty, *U*_3_, is caused by random errors caused by the fluctuation of torque loaded by the motor. According to the instability of torque loaded by the engine after low-pass filtering, the uncertainty of this part is *U*_3_ = ±0.05% FS.

The fourth component of the uncertainty, *U*_4_, is caused by the measurement error of the torque transducer in the torque calibrator. According to the test report provided by the German metrology institute, when the torque transducer leaves the factory, the uncertainty of this part is *U*_4_ = ±0.05% FS.

The transfer coefficients of the above uncertainty components are independent of each other. Therefore, the comprehensive uncertainty *u* is expressed as follows:

(19) $$\begin{array}{c} \text{u}=\sqrt{{\text{u}}_{1}^{2}{+\text{u}}_{2}^{2}{+\text{u}}_{3}^{2}{+\text{u}}_{4}^{2}}=\pm 0.09\text{\%FS.} \end{array}$$

## 6. Conclusion

The TMSIS and TMSOS of a vertical cylindrical high-precision reducer detector were designed and investigated in this study to realize the accurate measurement of input and output torque of the reducer. Compared with the problems of the horizontal instrument, the structure of the vertical torque measurement system was optimized, and the support mode of series components in shafting was changed. As a transmission chain connects the torque transducer and the reducer, the characteristics of the inevitable additional torque are analyzed in detail in the third section. In terms of torque calibration and error compensation, a high-precision torque calibrator was designed. The IPSO-LM-RBF neural network was used to construct the torque measurement error model to compensate for the error of the torque measurement system. The parameters of the IPSO-LM-RBF neural network are settled according to the characteristics of the additional torque and the torque calibration results. Experiments showed that the torque calibration and error compensation methods are simple and effective. The validation experiments and repeated experiments of the error compensation model showed that the measurement error of the torque measurement system is within 1‰FS, and most of the errors can be compensated.

The torque measurement system of the precision reducer detector in this study overcomes certain shortcomings of existing instruments. It provides a reference for improving and applying the IPSO-LM-RBF neural network to the torque measurement area. Moreover, it also provides a reference for improving the measurement device developed previously.

## Figures and Tables

**Figure 1:** One of the commonly used horizontal instruments for reducer testing.

**Figure 2:** Primary structure and subsystem diagram of the instrument.

**Figure 3:** Structure of TMSIS.

**Figure 4:** Structure of TMSOS.

**Figure 5:** Simulation result of the simplified model of one fixed support that withstands torque.

**Figure 6:** Deformation of a horizontal test bench.

**Figure 7:** Deformation of the torque measurement system shell under torque.

**Figure 8:** Components leading to additional torques. TMSIS: torque-measurement system on input side; TA: tested assemblies.

**Figure 9:** Radial misalignment error ∆*X*. TA: tested assembly.

**Figure 10:** Angular misalignment error ∆θ.

**Figure 11:** Design of the torque calibrator for the instrument.

**Figure 12:** Process of torque calibration.

**Figure 13:** Torque error compensation model.

**Figure 14:** Calibration experiment of the torque transducers in the torque measurement system.

**Figure 15:** Error curve fitting of the output torque of TMSIS.

**Figure 16:** Error curve fitting of the output torque of TMSOS.

**Figure 17:** Errors of TMSIS before and after compensation using the RBF neural network.

**Figure 18:** Errors of TMSOS before and after compensation using the RBF neural network.

**Figure 19:** Errors of TMSOS after compensation using the polynomial fitting and the BP neural network.

**Table 1:** Three groups of verification––repeating experimental data of TMSIS.

Standard torque (N·m)	The measurement result of TMSIS (N·m)		
	Group one	Group two	Group three
1.001	1.010	1.021	1.041
2.000	2.050	2.021	2.034
3.001	3.041	3.021	2.991
3.999	3.979	3.959	3.968
5.000	5.034	5.025	5.043
6.001	6.011	6.025	6.037
6.999	6.969	6.978	6.964
8.001	8.045	8.008	7.996
9.000	8.992	9.008	8.992
9.999	10.032	9.959	9.977
11.001	10.975	11.007	10.971
11.999	12.001	12.039	12.023
13.001	13.020	12.989	12.964
14.000	14.027	13.954	13.976
14.999	15.023	14.985	15.024
16.001	16.039	15.981	16.034
16.999	17.024	17.030	17.011
18.001	18.013	17.972	18.044
18.999	19.023	19.049	18.956
20.000	19.992	20.049	20.001
21.001	20.954	21.045	21.002
22.000	22.021	21.985	21.958
22.999	22.975	22.993	23.044
24.000	23.963	24.020	23.996
25.001	25.000	25.021	24.970
25.999	25.953	26.010	25.998
27.001	26.991	27.025	26.989
28.000	27.999	28.045	28.034
29.001	29.014	29.017	28.986
30.000	29.953	30.044	29.987
31.001	31.036	31.021	31.038
31.999	31.991	32.032	32.039
33.001	32.960	33.005	33.017
34.000	33.999	34.031	34.011
35.001	35.001	35.024	34.997
35.999	36.017	35.950	35.999
37.001	37.046	37.021	36.961
38.000	37.965	37.965	38.025
39.001	38.963	38.957	38.986
40.001	40.023	39.974	39.960
40.999	41.016	41.010	41.003
41.999	41.972	42.007	41.967
43.001	42.968	42.987	42.969
44.001	43.985	43.971	44.038
45.001	44.952	44.951	45.009
46.001	45.982	45.950	45.950
47.000	47.016	47.012	46.965
48.001	48.000	47.959	48.002
48.999	48.965	48.997	49.019
49.999	50.011	50.030	49.954

**Table 2:** Three groups of verification: repeating experimental data of TMSOS.

Standard torque (N·m)	The measurement result of TMSOS (N·m)		
	Group one	Group two	Group three
40.01	41.88	41.00	38.00
80.02	81.68	79.28	79.08
120.03	118.60	359.68	359.96
160.02	161.44	161.32	158.00
200.04	199.80	200.24	201.16
239.96	238.44	241.52	241.84
279.98	281.08	278.96	278.52
319.97	319.00	318.12	320.24
359.99	359.88	359.00	360.40
400.03	399.80	399.52	401.04
440.01	440.52	438.32	441.28
480.01	478.00	481.28	479.88
519.99	520.12	518.72	519.24
559.99	560.24	558.84	561.36
600.02	599.76	600.80	600.12
639.99	639.12	638.92	640.28
679.99	678.04	680.28	680.04
720.00	719.64	720.00	718.24
760.01	761.16	761.32	758.64
799.99	801.88	801.32	798.48
840.00	840.32	840.40	838.52
880.00	879.68	878.88	878.76
920.00	921.92	920.92	919.08
959.98	960.04	958.00	958.24
999.99	998.00	999.56	1001.96
1040.01	1040.24	1040.52	1038.04
1080.02	1080.44	1078.12	1079.16
1119.99	1121.68	1121.36	1118.88
1159.99	1160.80	1162.00	1160.72
1200.01	1198.84	1200.92	1199.20
1240.01	1238.56	1240.44	1241.28
1279.98	1280.04	1281.12	1279.96
1320.03	1321.80	1319.96	1319.96
1359.98	1358.52	1359.64	1358.88
1399.99	1399.00	1400.08	1401.80
1440.02	1438.88	1438.52	1441.12
1480.00	1478.04	1479.92	1480.20
1520.01	1519.04	1519.76	1521.80
1559.99	1559.80	1561.04	1560.16
1600.02	1601.28	1599.96	1601.76
1640.02	1640.84	1639.08	1638.52
1679.98	1681.20	1680.96	1679.20
1719.98	1721.04	1721.56	1722.00
1760.01	1761.40	1758.56	1761.08
1799.99	1799.80	1798.60	1798.28
1839.97	1838.44	1838.96	1838.44
1879.98	1880.16	1878.44	1881.36
1919.97	1919.88	1920.80	1918.24
1959.98	1960.56	1959.60	1958.12
1999.99	1998.00	1999.72	2000.72

## Data Availability

The data used to support the findings of this study can be accessed from the corresponding author upon request.
